# Relationship between serum TGF- β 1, MMP-9 and IL-1β and pathological features and prognosis in breast cancer

This article has been retracted.

**DOI:** 10.3389/fgene.2022.1095338

**Published:** 2023-01-12

**Authors:** Shuyan Cai, Jianwei Zheng, Huimin Song, Haoliang Wu, Wang Cai

**Affiliations:** Department of General Surgery, Beijing Chaoyang Hospital Affiliated with Capital Medical University, Beijing, China

**Keywords:** breast cancer, pathological features, transforming growth factor-β 1, matrix metalloproteinase-9, interleukin-1 β, prognosis, correlation

## Abstract

To investigate the levels of serum transforming growth factor-β 1 (TGF-β1), Matrix metalloproteinase-9 (MMP-9) and Interleukin-1 β (IL-1 β) in breast cancer (BC), and analyzing their relationship with pathological features and prognosis. Retrospective analysis of 86 subjects with BC (BC subgroup) and another 50 healthy subjects (control subgroup) during the same period were included. The clinical data were collected. In this research, in BC subgroup, The levels of serum TGF- β 1, MMP-9 and IL-1 β were significantly higher than those in control subgroup. The levels of TGF- β 1 and MMP-9 in serum of BC subjects was correlated with clinical stage, histological grade, lymph node metastasis and molecular classification, but not with age, tumor size and menopausal status. The level of serum IL-1 β was related to tumor size, clinical stage, histological grade and lymph node metastasis. Multivariate Logistic regression analysis showed that the high level of serum TGF- β1 and MMP-9 was independent risk factors for BC. High level of serum IL-1 β was not an independent risk factor for BC. The 3-year disease-free survival rate in high TGF- β1 subgroup and high MMP-9 subgroup was significantly lower than that in low TGF- β 1 subgroup and low MMP- 9 subgroup. To conclude, serum TGF- β 1, MMP-9 and IL-1β are highly expressed in BC, and the subjects with elevated serum levels of TGF- β 1 and MMP-9 suggests poor prognosis.

## Introduction

Breast cancer (BC) is a high incidence of malignant tumor in the world, which seriously affects the safety and quality of life of women (Ghoncheh et al., 2016). A study (Bray et al., 2018) shows that tumor metastasis is the main causes of death in subjects with BC. Understanding its mechanism is helpful to find new treatment targets and guide clinical accurate treatment. Transforming growth factor-β 1 (TGF-β 1) is a polypeptide encoded by genes on human chromosome 19. Almost all cells in human body can synthesize TGF-β 1, which has the functions of immune regulation, promoting cell growth and differentiation, angiogenesis, immune regulation and so on (Desai et al., 2018). Some studies (Narod et al., 2015; Zheng et al., 2020; Chandra Jena et al., 2021; Xia et al., 2022) have found that under normal physiological conditions, TGF- β 1 inhibits the growth of tumor cells, and this inhibition still exists in the early stage of tumor, but once tumor cells enter the uncontrollable growth stage, the inhibition of TGF- β 1 will turn into promoting effect, leading to tumor occurrence and development. At present, related studies (Zhang et al., 2014, 7; Labrèche et al., 2021) have corroborated that BC-associated fibroblasts (CAFs) and epithelial-mesenchymal transformation (EMT) are the key links of tumor cell proliferation and metastasis. TGF-β 1 can induce CAFs formation and promote tumor cell proliferation. EMT is closely related to extracellular matrix (ECM) remodeling. Matrix metalloproteinases (MMPs) are a kind of proteolytic enzymes, whose main function is to degrade ECM. MMP-9 is a member of the MMPs family, also known as gelatinase, which can degrade gelatin, type IV collagen and type V collagen in ECM, thus destroying the structure of ECM, inducing EMT, and promoting tumor cell invasion and metastasis (Heintz and Meyer-Schwesinger, 2021). Other studies (Lazaar and Panettieri, 2005; Khodabakhshi et al., 2021) have shown that interleukin-1 β (IL-1 β) plays an important role in tumor growth, proliferation, invasion and metastasis. Its high expression can lead to inflammatory cascade reaction and promote tumor angiogenesis. At present, there are few studies on the relationship between the levels of serum TGF- β 1, MMP-9, IL-1 β and pathological features and prognosis of BC. In recent years, biomarkers have been used as a tool in the diagnosis and treatment of cancer, which has become a new direction of cancer research and has higher value for cancer screening and guiding clinical treatment. In view of the above research basis, we evaluated the relationship between the expression of serum TGF- β 1, MMP-9 and pathological features and prognosis of breast cancer. The clinical data of 86 patients with breast cancer and 50 healthy subjects in the same period were retrospectively analyzed. The levels of serum TGF- β 1 and MMP-9 were detected, and the relationship between the expression of TGF- β 1, MMP-9 and pathological characteristics of patients was analyzed. The relationship between the expression of TGF- β 1, MMP-9 and survival and prognosis was analyzed by Kaplan-Meier method.

### General information of patients

86 subjects with BC (BC subgroup) treated in our hospital from March 2016 to March 2019 were selected retrospectively. Inclusion criteria: 1) Age ≥18 years old; 2) BC diagnosed by pathology and first onset; 3) Expected survival time ≥6 months. Exclusion criteria: 1) Subjects merged with other malignant tumors; 2) Subjects with hematological diseases; 3) Subjects merged with acute and chronic infection. Another 50 healthy subjects in the same period were selected as the control subgroup.

### Clinical data collection

The age, tumor size, clinical stage, lymph node metastasis, histological grade, molecular classification and menopause of BC subjects were collected by professionals.

## Serum TGF- β 1, MMP-9, and IL-1β levels detection

The serum samples of subjects with BC before operation or before chemotherapy were collected, and the fasting venous blood of healthy subjects in the morning was collected. The levels of TGF- β 1, MMP-9 and IL-1β in serum were estimated by enzyme linked immunosorbent assay (ELISA). The operation was carried out strictly according to the instructions of the kit.

### Follow-up

The subjects were followed up for 36 months by outpatient reexamination and telephone follow-up, and the progression-free survival time was recorded.

### Observation indicators

1) Serum TGF- β 1, MMP-9, and IL-1β levels in BC subgroup and control subgroup. 2) The relationship between serum TGF- β 1, MMP-9, IL-1β, and clinicopathological features. 3) The 3-year disease-free survival rate of different TGF- β 1 and MMP-9 level subgroups.

## Data statistics

The data were analyzed by SPSS 24.0. The measurement data of this test were tested for normality and homogeneity of variance. Single factor ANOVA was used to conform to the data of normal distribution and homogeneity of variance. Which was expressed by (‾*x* ± *s*). LSD method was used for pairwise comparison among groups. The counting data were expressed by [n (%)] and tested by χ^2^. The relationship between serum TGF- β 1, MMP-9, IL-1β and clinicopathological features was analyzed by Logistic regression analysis, survival curve was drawn by Kaplan-Meier method, and Log-Rank χ^2^ test was used. The difference was statistically significant (*p* < 0.05).

## Results

### Serum levels of TGF- β 1, MMP-9 and IL-1β

The levels of serum TGF- β 1, MMP-9 and IL-1β in BC subgroup (TGF-β1: 27.18 ± 6.24, MMP-9: 73.17 ± 12.84, IL-1β: 132.86 ± 40.43) were significantly higher than those in control subgroup (TGF-β1: 13.45 ± 4.36, MMP-9: 18.91 ± 5.70, IL-1β: 40.17 ± 3.86) (*p* < 0.05). As corroborated in Table 1; Figures 1A–C.

**TABLE 1:** Comparison of serum TGF- β 1, MMP-9 and IL-1β levels between the two subgroups (‾*x* ± *s*).

Groups	n	TGF-β1 (µg/ml)	MMP-9 (ng/ml)	IL-1β (ng/L)
The BC subgroup	86	27.18 ± 6.24	73.17 ± 12.84	132.86 ± 40.43
The control subgroup	50	13.45 ± 4.36	18.91 ± 5.70	40.17 ± 3.86
*t*		13.723	28.272	16.144
*P*		<0.001	<0.001	<0.001

**FIGURE 1:** Serum **(A)** TGF-β1, **(B)** MMP-9 and **(C)** IL-1β levels between the two subgroups.

### The relationship between serum TGF- β, 1, MMP-9, IL-1β levels and pathological features in subjects with BC

The relationship between serum TGF-β1, MMP-9 levels was correlated with clinical stage (TGF-β1: t = 2.196, *p* = 0.031; MMP-9: t = 2.003,*p* = 0.048), histological grade (TGF-β1: t = 3.336, *p* = 0.001; MMP-9: t = 2.249,*p* = 0.027), lymph node metastasis (TGF-β1: t = 3.399, *p* = 0.001; MMP-9: t = 2.308,*p* = 0.023) and molecular classification (TGF-β1: F = 4.201, *p* = 0.005; MMP-9: F = 2.796,*p* = 0.034) (*p* < 0.05), but not with age (TGF-β1: t = 0.893, *p* = 0.374; MMP-9: t = 0.723,*p* = 0.374), tumor size (TGF-β1: t = 0.655, *p* = 0.514; MMP-9: t = 0.080,*p* = 0.937) and menopause (TGF-β1: t = 0.217, *p* = 0.828; MMP-9: t = 0.862,*p* = 0.391) (*p* > 0.05). Serum IL-1 β in patients with BC was correlated with tumor size (t = 2.106, *p* = 0.038), clinical stage (t = 2.607, *p* = 0.011), histological grade (t = 2.975, *p* = 0.004) and lymph node metastasis (t = 2.955, *p* = 0.004) (*p* < 0.05), but not with age (t = 0.437, *p* = 0.664), molecular classification (F = 2.315, *p* = 0.386) and menopausal state (*t* = 1.067, *p* = 0.289) (*p* > 0.05) (Table 2; Figures 2A–C).

**TABLE 2:** Comparison of serum TGF- β 1,MMP-9 and IL-1 β levels in subjects with BC with different pathological features.

Clinicopathological features	n	TGF-β1	t/F	P	MMP-9	t/F	P	IL-1β	t/F	P
Age (years)										
<50	32	27.91 ± 6.04	0.893	0.374	72.17 ± 10.33	0.723	0.472	130.40 ± 38.51	0.437	0.664
≥50	54	26.75 ± 5.69			73.76 ± 9.58			134.32 ± 41.24		
Tumor size (cm)										
≤3	36	26.68 ± 5.70	0.655	0.514	73.06 ± 10.64	0.080	0.937	122.59 ± 35.14	2.106	0.038
>3	50	27.54 ± 6.21			73.25 ± 11.08			140.25 ± 40.50		
Clinical stage										
Stage I ∼ II	21	25.08 ± 4.36	2.196	0.031	69.05 ± 12.27	2.003	0.048	115.33 ± 34.54	2.607	0.011
Stage III ∼ IV	65	27.86 ± 5.24			74.50 ± 10.35			138.52 ± 35.72		
Histological grade										
Stage I ∼ II	42	25.37 ± 4.87	3.336	0.001	70.81 ± 9.25	2.249	0.027	120.37 ± 37.10	2.975	0.004
Stage III	44	28.91 ± 5.02			75.42 ± 9.74			144.78 ± 38.91		
Lymph node metastasis										
Yes	30	29.15 ± 4.36	3.399	0.001	76.24 ± 9.31	2.308	0.023	147.38 ± 32.65	2.955	0.004
No	56	26.12 ± 3.70			71.53 ± 8.86			125.08 ± 33.72		
Molecular classification										
LA type	11	24.53 ± 4.48	4.201	0.005	69.03 ± 8.81	2.796	0.034	129.35 ± 37.15	2.315	0.386
LB type	34	25.10 ± 4.22			70.26 ± 9.47			131.73 ± 38.20		
TNBC type	15	32.73 ± 3.46			76.30 ± 8.73			135.14 ± 35.69		
HER-2 type	26	27.80 ± 3.71			76.92 ± 8.54			134.51 ± 36.07		
Menopausal state										
Menopause	41	27.05 ± 5.21	0.217	0.828	74.05 ± 9.27	0.862	0.391	137.65 ± 39.24	1.067	0.289
Premenopausal	45	27.30 ± 5.43			72.37 ± 8.80			128.50 ± 40.13		

**FIGURE 2:** Serum **(A)** TGF-β1, **(B)** MMP-9 and **(C)** IL-1β levels in subjects with BC with different pathological features.

### Risk assessment of BC by TGF- β 1 and MMP-9

Univariate analysis showed that serum TGF- β 1, MMP-9 and IL-1 β were influencing factors of BC (*p* < 0.05), while multivariate analysis showed that high level of serum TGF- β 1 and MMP-9 were independent risk factors of BC (*p* < 0.05), serum IL-1 β was not an independent risk factor for BC (*p* > 0.05). As corroborated in Table 3.

**TABLE 3:** Predictive value of serum TGF- β 1, MMP-9 and IL-1 β in BC.

Serum index	Single factor analysis		Multi-factor analysis	
	OR (95%CI)	P	OR (95%CI)	P
TGF-β1	2.68 (1.27–3.94)	<0.001	1.73 (1.15–3.18)	0.005
MMP-9	3.57 (1.49–4.12)	<0.001	2.16 (1.88–3.21)	<0.001
IL-1 β	1.74 (0.91–2.56)	0.045	1.22 (0.78–2.03)	0.089
Age	0.95 (0.73–2.07)	0.357	1.03 (0.78–1.67)	0.442
Tumor size	1.09 (0.82–1.95)	0.318	1.12 (0.85–1.94)	0.371
Menopausal state	1.46 (1.09–2.53)	0.116	1.24 (0.87–1.85)	0.255

### Relationship between serum TGF- β 1, MMP-9 levels and prognosis in subjects with BC

86 subjects with BC were divided into high level subgroup and low level subgroup according to the median of serum TGF- β 1 and MMP-9 levels. The results showed that the 3-year disease-free survival rate of high TGF- β 1 subgroup (69.00%) and high MMP-9 level subgroup (61.90%) was significantly lower than that of low TGF- β 1 subgroup (86.40%) and low MMP-9 level subgroup (84.11%) (*p* < 0.05), as corroborated in Figures 3, 4.

**FIGURE 3:** Survival curve of subjects with different serum TGF- β 1 level.

**FIGURE 4:** Survival curve of subjects with different serum MMP-9 level.

## Discussion

According to the epidemiological survey (Azamjah et al., 2019), the incidence and mortality of female BC in China are 36.1/10^5^ and 8.8/10^5^ respectively. Although the overall level is relatively low, China has a large population base, and the number of morbidity and mortality still ranks first in the world, which should be paid attention to. The global cancer survival analysis report (Morey et al., 2019) shows that early cancer is easier to treat than advanced subjects, and subjects are more likely to survive. Therefore, it is of great significance for the prevention and treatment of BC to understand the mechanism of progression and metastasis of BC and to identify the risk factors related to BC.

The results of this study showed that the levels of serum TGF- β 1, MMP-9 and IL-1 β in BC subjects were significantly higher than those in healthy controls, suggesting that serum TGF- β 1, MMP-9 and IL-1 β were highly expressed in subjects with BC, which may be involved in the development of BC. TGF- β 1 plays a dual role in tumorigenesis and development, and inhibits tumor cells in the early stage of carcinogenesis. When entering the tumor progression stage, the inhibitory effect of TGF- β 1 will disappear, and these tumor cells begin to secrete a large amount of TGF- β 1, which plays a promoting role (Liu et al., 2016; Caja et al., 2018). Previous study (Hiensch et al., 2021) has corroborated that the level of serum TGF- β 1 in subjects with BC is higher than that in subjects with benign breast lesions and healthy women. Existing evidence shows that ECM remodeling is an important process of invasion and metastasis of breast tumor cells. MMP-9 is an important gelatinase in MMPs, which can degrade ECM on the surface of tumor, destroy the physical barrier of basement membrane, and cause tumor cells to rush to the surrounding tissue without barrier (Liao et al., 2019). A large number of reports (Liu et al., 2017; Joseph et al., 2020) have shown that MMP-9 is highly expressed in BC tissues and is closely related to tumor metastasis. Whereas, inflammatory factors can induce breast cancer cell EMT and promote tumor cell metastasis.

This study found that serum TGF- β 1 and MMP-9 levels were higher in subjects with clinical II ∼ IV stage, histological grade III, with lymph node metastasis and TNBC type BC. There was no significant difference in serum TGF- β 1 and MMP-9 levels among subjects with different age, tumor size and menopausal status, indicating that the levels of TGF- β 1 and MMP-9 were related to clinical stage, histological grade, lymph node metastasis and molecular classification of BC. Studies (Tong et al., 2019; Huang et al., 2021) have corroborated that TGF- β 1 can participate in the development of BC by inducing or inhibiting autophagy and apoptosis. The higher the level is, the more significant the change of related signal pathway is, the faster the tumor progression is and the higher the malignant degree is. MMP-9 plays an important role in remodeling tumor microenvironment, and tumor-associated macrophages also secrete MMP-9, and its level can reflect the malignant degree and prognosis of tumor (Shi et al., 2017; Mondal et al., 2020, 9). BC has high heterogeneity, and the prognosis is different according to different molecular classifications. The prognosis of subjects with TNBC type is worse than that of LA type, LB type and HER- 2 type (Goldhirsch et al., 2013; Badr et al., 2018). This is because all hormone receptors in subjects with TNBC type are negative, there is no specific therapy target, the degree of malignancy is high, and the prognosis is poor (López-Ozuna et al., 2016). Further Logistic regression analysis also showed that the high level of TGF- β 1 and MMP-9 was an independent risk factor for BC, which confirmed that TGF- β 1 and MMP-9 were involved in the invasion and metastasis of BC. In this study, the level of serum IL-1 β was related to tumor size, clinical stage, histological grade and lymph node metastasis, but Logistic regression analysis showed that IL-1 β was not an independent risk factor for BC. In spite of this, inflammatory factors (including IL-1 β) are involved in the mechanism of tumor development, but there are many factors leading to inflammatory response, such as tissue injury, infection and so on. The increase of IL- β alone is of little significance in predicting breast cancer, and other indexes need to be combined (Blevins et al., 2015).

The ultimate goal of antineoplastic therapy is to prolong the survival time of subjects and improve the quality of life. A survey on the 5-year survival rate of BC subjects in the United States (Morey et al., 2019) shows that the 5-year survival rates of stage I, II, III and IV BC subjects are 98%, 92%, 75%, and 27%, respectively, indicating that the higher the clinical stage, the lower the survival rate and the worse the prognosis. In this study, 3-year follow-up showed that the 3-year disease-free survival rate of high TGF- β 1 and MMP-9 subgroup was lower than that of low TGF- β 1 and MMP-9 subgroup, suggesting that there is a certain relationship between the level of serum TGF- β 1 and MMP-9 and prognosis of subjects with BC, which can be used as one of the indexes to judge the prognosis of subjects with BC.

## Limitations

In addition, clinical multi center and large sample experiments are needed to further verify the conclusions of this study. The relationship among TGF- β 1, MMP-9 and IL-1 β and the value of combined use in the diagnosis of breast cancer need to be confirmed by further study.

## Conclusion

To sum up, the levels of serum TGF- β 1, MMP-9 and IL-1 β in subjects with BC are increased, and the levels of TGF- β 1 and MMP-9 are related to clinical stage, lymph node metastasis, histological grade and molecular classification, which can effectively predict the prognosis of subjects.

## Data Availability

The original contributions presented in the study are included in the article/supplementary material, further inquiries can be directed to the corresponding author.

## References

[B1] AzamjahN.Soltan-ZadehY.ZayeriF. (2019). Global trend of breast cancer mortality rate: A 25-year study. Asian Pac J. Cancer Prev. 20, 2015–2020. 10.31557/APJCP.2019.20.7.2015 31350959 PMC6745227

[B2] BadrL. K.BourdeanuL.AlatrashM.BekarianG. (2018). Breast cancer risk factors: A cross- cultural comparison between the west and the east. Asian Pac J. Cancer Prev. 19, 2109–2116. 10.22034/APJCP.2018.19.8.2109 30139209 PMC6171412

[B3] BlevinsM. A.TowersC. G.PatrickA. N.ZhaoR.FordH. L. (2015). The SIX1-EYA transcriptional complex as a therapeutic target in cancer. Expert Opin. Ther. Targets 19, 213–225. 10.1517/14728222.2014.978860 25555392 PMC4336540

[B4] BrayF.FerlayJ.SoerjomataramI.SiegelR. L.TorreL. A.JemalA. (2018). Global cancer statistics 2018: GLOBOCAN estimates of incidence and mortality worldwide for 36 cancers in 185 countries. CA Cancer J. Clin. 68, 394–424. 10.3322/caac.21492 30207593

[B5] CajaL.DituriF.MancarellaS.Caballero-DiazD.MoustakasA.GiannelliG. (2018). TGF-Β and the tissue microenvironment: Relevance in fibrosis and cancer. Int. J. Mol. Sci. 19, E1294. 10.3390/ijms19051294 PMC598360429701666

[B6] Chandra JenaB.Kanta DasC.BanerjeeI.DasS.BharadwajD.MajumderR. (2021). Paracrine TGF-β1 from breast cancer contributes to chemoresistance in cancer associated fibroblasts via upregulation of the p44/42 MAPK signaling pathway. Biochem. Pharmacol. 186, 114474. 10.1016/j.bcp.2021.114474 33607074

[B7] DesaiA. A.JimenezR. E.HoskinT. L.DayC. N.BougheyJ. C.HiekenT. J. (2018). Treatment outcomes for pleomorphic lobular carcinoma *in situ* of the breast. Ann. Surg. Oncol. 25, 3064–3068. 10.1245/s10434-018-6591-6 29947004

[B8] GhonchehM.PournamdarZ.SalehiniyaH. (2016). Incidence and mortality and epidemiology of breast cancer in the world. Asian Pac J. Cancer Prev. 17, 43–46. 10.7314/apjcp.2016.17.s3.43 27165206

[B9] GoldhirschA.WinerE. P.CoatesA. S.GelberR. D.Piccart-GebhartM.ThürlimannB. (2013). Personalizing the treatment of women with early breast cancer: Highlights of the st gallen international expert consensus on the primary therapy of early breast cancer 2013. Ann. Oncol. 24, 2206–2223. 10.1093/annonc/mdt303 23917950 PMC3755334

[B10] HeintzL.Meyer-SchwesingerC. (2021). The intertwining of autophagy and the ubiquitin proteasome system in podocyte (Patho)Physiology. Cell. Physiol. Biochem. 55, 68–95. 10.33594/000000432 34523304

[B11] HienschA. E.MijwelS.BargielaD.WengströmY.MayA. M.RundqvistH. (2021). Inflammation mediates exercise effects on fatigue in patients with breast cancer. Med. Sci. Sports Exerc 53, 496–504. 10.1249/MSS.0000000000002490 32910094 PMC7886356

[B12] HuangM.FuM.WangJ.XiaC.ZhangH.XiongY. (2021). TGF-β1-activated cancer-associated fibroblasts promote breast cancer invasion, metastasis and epithelial-mesenchymal transition by autophagy or overexpression of FAP-α. Biochem. Pharmacol. 188, 114527. 10.1016/j.bcp.2021.114527 33741330

[B13] JosephC.AlsaleemM.OrahN.NarasimhaP. L.MiligyI. M.KurozumiS. (2020). Elevated MMP9 expression in breast cancer is a predictor of shorter patient survival. Breast Cancer Res. Treat. 182, 267–282. 10.1007/s10549-020-05670-x 32445177 PMC7297818

[B14] KhodabakhshiA.AkbariM. E.MirzaeiH. R.SeyfriedT. N.KalamianM.DavoodiS. H. (2021). Effects of ketogenic metabolic therapy on patients with breast cancer: A randomized controlled clinical trial. Clin. Nutr. 40, 751–758. 10.1016/j.clnu.2020.06.028 32703721

[B15] LabrècheC.CookD. P.Abou-HamadJ.PascoalJ.PryceB. R.Al-ZahraniK. N. (2021). Periostin gene expression in neu-positive breast cancer cells is regulated by a FGFR signaling cross talk with TGFβ/PI3K/AKT pathways. Breast Cancer Res. 23, 107. 10.1186/s13058-021-01487-8 34809697 PMC8607680

[B16] LazaarA. L.PanettieriR. A. (2005). Airway smooth muscle: A modulator of airway remodeling in asthma. J. Allergy Clin. Immunol. 116, 488–495. quiz 496. 10.1016/j.jaci.2005.06.030 16159613

[B17] LiaoS.-J.LuoJ.LiD.ZhouY.-H.YanB.WeiJ.-J. (2019). TGF-β1 and TNF-α synergistically induce epithelial to mesenchymal transition of breast cancer cells by enhancing TAK1 activation. J. Cell. Commun. Signal 13, 369–380. 10.1007/s12079-019-00508-8 30739244 PMC6732143

[B18] LiuF.-L.MoE.-P.YangL.DuJ.WangH.-S.ZhangH. (2016). Autophagy is involved in TGF-β1-induced protective mechanisms and formation of cancer-associated fibroblasts phenotype in tumor microenvironment. Oncotarget 7, 4122–4141. 10.18632/oncotarget.6702 26716641 PMC4826194

[B19] LiuY.LvH.WuX.ZhouJ.ShiY.WenJ. (2017). Demethylation of repressor element-1 silencing transcription (REST) suppresses the malignant phenotype of breast cancer via MMP9. Oncol. Res. 25, 445–454. 10.3727/096504016X14747368729786 27697091 PMC7841195

[B20] López-OzunaV. M.HachimI. Y.HachimM. Y.LebrunJ.-J.AliS. (2016). Prolactin pro-differentiation pathway in triple negative breast cancer: Impact on prognosis and potential therapy. Sci. Rep. 6, 30934. 10.1038/srep30934 27480353 PMC4969612

[B21] MondalS.AdhikariN.BanerjeeS.AminS. A.JhaT. (2020). Matrix metalloproteinase-9 (MMP-9) and its inhibitors in cancer: A minireview. Eur. J. Med. Chem. 194, 112260. 10.1016/j.ejmech.2020.112260 32224379

[B22] MoreyB. N.GeeG. C.von EhrensteinO. S.Shariff-MarcoS.CancholaA. J.YangJ. (2019). Higher breast cancer risk among immigrant asian American women than among US-born asian American women. Prev. Chronic Dis. 16, E20. 10.5888/pcd16.180221 30767860 PMC6395083

[B23] NarodS. A.IqbalJ.GiannakeasV.SopikV.SunP. (2015). Breast cancer mortality after a diagnosis of ductal carcinoma *in situ* . JAMA Oncol. 1, 888–896. 10.1001/jamaoncol.2015.2510 26291673

[B24] ShiZ. M.LiuY. N.FuB.ShenY. F.LiL. M. (2017). Expression profile of eukaryotic translation initiation factor and matrix metalloproteinase 9 in endometrial cancer tissue. J. Biol. Regul. Homeost. Agents 31, 1053. 10.23812/21-128-L 29254314

[B25] TongH.YinH.HossainM. A.WangY.WuF.DongX. (2019). Starvation-induced autophagy promotes the invasion and migration of human bladder cancer cells via TGF-β1/Smad3-mediated epithelial-mesenchymal transition activation. J. Cell. Biochem. 120, 5118–5127. 10.1002/jcb.27788 30320898

[B26] XiaF.LiQ.LuoX.WuJ. (2022). Association between urinary metals and leukocyte telomere length involving an artificial neural network prediction: Findings based on NHANES 1999-2002. Front. Public Health 10, 963138. 10.3389/fpubh.2022.963138 36172207 PMC9511050

[B27] ZhangH.CaiK.WangJ.WangX.ChengK.ShiF. (2014). MiR-7, inhibited indirectly by lincRNA HOTAIR, directly inhibits SETDB1 and reverses the EMT of breast cancer stem cells by downregulating the STAT3 pathway. Stem Cells 32, 2858–2868. 10.1002/stem.1795 25070049

[B28] ZhengX.ShiJ.WuJ. (2020). Analysis of factors and corresponding interactions influencing clinical management assistant ability using competency model in China. Med. Baltim. 99 (51), e23516. 10.1097/MD.0000000000023516 PMC774818533371073

